# Evaluation of Multimedia Courseware-Assisted Teaching Effect of Medical Images Based on the Deep Learning Algorithm

This article has been retracted.

**DOI:** 10.1155/2022/5991087

**Published:** 2022-09-29

**Authors:** Yu-Na Chen, Xuesen Zhang

**Affiliations:** ^1^Department of Medical Technology, Shangqiu Medical College, Shangqiu 476100, Henan, China; ^2^School of Economics and Management, Anhui University of Science and Technology, Huainan, Anhui, China

## Abstract

In order to improve the dynamic evaluation ability of medical image multimedia courseware-assisted teaching effect, the evaluation of medical image multimedia courseware-assisted teaching effect based on a deep learning algorithm is proposed. The statistical data analysis model of medical image multimedia courseware-assisted teaching effect is established to estimate its utilization rate and scale parameters. Based on the prediction of spatial attribute parameters, the classification big data mining model of medical image multimedia courseware-assisted teaching is constructed by using the deep learning algorithm, mining association rules and frequent item sets that can dynamically reflect the quality of medical image multimedia courseware-assisted teaching, and extracting the statistical feature of the dataset of constraint indicators of medical image multimedia courseware-assisted teaching effect to improve the teaching quality of medical imaging course. The simulation results show that this method has a better precision delivery effect, higher dynamic matching degree of teaching evaluation parameters, more than 90% reliability, and better clustering of statistical eigenvalues.

## 1. Introduction

Through the evaluation of the effect of medical image multimedia courseware-assisted teaching, combined with the analysis of the use characteristics of medical image multimedia courseware-assisted teaching, it is necessary to evaluate the effect of medical image multimedia courseware-assisted teaching under the multisource information resource as a service (miraas) mode so as to improve the intelligent service level of medical image multimedia courseware-assisted teaching [1, 2].

The research on the evaluation of the effect of medical image multimedia courseware-assisted instruction is realized by analyzing the utilization state characteristics of medical image multimedia courseware-assisted instruction [3, 4] and analyzing the data quantification index parameters. In the traditional methods, the attribute parameter analysis of the auxiliary teaching evaluation of medical image multimedia courseware is realized through coordinate convolution information fusion and remote sensing resolution control [5]. Currently, the multimedia resource management method of medical image multimedia courseware auxiliary teaching based on statistical feature extraction [6] is adopted to establish a data classification detection model to realize the auxiliary teaching effect evaluation of medical image multimedia courseware. However, the fusion degree and sharing level of traditional methods for medical image multimedia courseware-assisted teaching effect evaluation are not high. Through multisource remote sensing parameter analysis, combined with high-standard medical image multimedia courseware-assisted teaching construction feature parameter fusion, the medical image multimedia courseware-assisted teaching effect evaluation is realized. However, the traditional methods have low evaluation accuracy and large calculation cost.

In view of the above problems, this paper proposes an evaluation method of medical image multimedia courseware assistant teaching effect based on the deep learning algorithm. It shows the superiority of this method in improving the evaluation ability of medical image multimedia courseware. Finally, the simulation test analysis shows the superiority of this method in improving the teaching effect of medical image multimedia courseware.

## 2. Deep Learning Algorithm Theory

Deep learning is to learn the inherent rules and representation levels of sample data. The information obtained in the learning process is of great help to the interpretation of data such as words, images, and sounds [7, 8]. The ultimate goal of deep learning is to enable machines to have analytical learning ability like people and to recognize data such as words, images, and sounds. Deep learning is a complex machine learning algorithm, and its effect on speech and image recognition is far superior to the previously related technologies. Deep learning has made many achievements in search technology, data mining, machine learning, machine translation, natural language processing, multimedia learning, voice, recommendation, personalization technology, and other related fields [9, 10]. Deep learning has made great achievements in search technology, data mining, machine learning, machine translation, natural language processing, multimedia learning, and other related fields. Deep learning is a general term for a class of pattern analysis methods. As far as the specific research content is concerned, it mainly involves three kinds of methods: convolutional neural network, sparse coding, and deep confidence network [11, 12]. After the initial “low-level” feature representation is gradually transformed into a “high-level” feature representation through multilevel processing, complex learning tasks such as classification can be completed with a “simple model”. Therefore, deep learning can be understood as “feature learning” or “representation learning.” Deep learning is a kind of machine learning, and machine learning is the only way to realize artificial intelligence. The concept of deep learning originates from the research of artificial neural networks, and the multilayer perceptron with multiple hidden layers is a deep learning structure. Deep learning forms more abstract high-level representation attribute categories or features by combining low-level features to discover distributed feature representations of data. The calculation involved in deep learning to generate an output from an input can be represented by a flow chart. The depth of the structure usually has 3, 6, or even 10 layers of hidden nodes, as shown in Figure 1.

Each node in the deep learning model represents a basic calculation and a calculated value, and the calculated result is applied to the values of the child nodes of this node. We consider a computational set, which can be allowed in every node and possible graph structure, and define a family of functions. The input node has no parent node, and the output node has no child nodes. Through layer-by-layer feature transformation, the feature representation of the sample in the original space is transformed into a new feature space, thus making classification or prediction easier. Compared with the method of constructing features by artificial rules, using big data to learn features can better depict the rich internal information of data.

## 3. Overall Structure Design and Modular Analysis of Medical Multimedia Courseware-Aided Teaching Effect Evaluation System

### 3.1. Overall Framework

The networked control technology of the Internet of things is used to realize the networked control of the process of medical image multimedia courseware-assisted teaching effect evaluation. The constructed medical image multimedia courseware-assisted teaching effect evaluation system includes an information collection module, a data analysis module, and a resource scheduling module. The data bus development platform of the medical image multimedia courseware-assisted teaching effect evaluation system is established. The utilization rate and scale parameters of the medical image multimedia courseware-assisted teaching effect are estimated [13, 14]. The standard IEEE interface protocol is adopted to realize the component management, data management, and report management of resource information of the medical image multimedia courseware-assisted teaching effect evaluation system. The medical image multimedia courseware is the standardized content of the auxiliary teaching system, so it has the following characteristics:

1. The design of medical image multimedia courseware-aided teaching system is to apply the system method to study and explore the essential relationship between each element in the teaching and learning system and between the element and the whole and comprehensively consider and coordinate their relations in the design so that each element can be organically combined to complete the function of the teaching system. If we do not consider the various elements that affect the implementation of the solution and the relationship between them, the designed solution will not achieve its expected goals.
2. The research object of teaching system design is the system of learning and teaching at different levels. This system includes the contents, conditions, resources, methods, and activities to promote students' learning. The process of teaching system design is the process of making specific plans for these elements that affect the teaching effect.
3. The purpose of teaching system design is to transform the principles and methods of basic theories such as learning theory and teaching theory into solutions to practical teaching problems. It is to creatively solve problems in teaching by using known teaching laws. The results or products of teaching system design are verified teaching system implementation plans that can achieve the expected functions, including teaching objectives, teaching activities, and implementation plans required to achieve certain teaching objectives and relevant supporting materials.

Based on the principles of intensive construction, coconstruction and sharing, overall planning and promotion, the evaluation system of medical image multimedia courseware-assisted teaching effect is constructed. The overall structure of the system is shown in Figure 2.

The web framework system is adopted to evaluate and optimize the effect of medical image multimedia courseware-assisted teaching under multimedia technology. The image teaching is the main content, the advanced client-server system is selected, the switching fast Ethernet technology and the relevant supporting network equipment are applied, and the star topology structure and integrated wiring technology are adopted to realize the automatic control of the evaluation of medical image multimedia courseware-assisted teaching effect, The network design of the system is shown in Figure 3.

### 3.2. Statistical Dataset of Medical Multimedia Courseware-Assisted Teaching Effect

In order to evaluate the teaching effect of medical image multimedia courseware based on the deep learning algorithm, first, a statistical data analysis model of medical image multimedia courseware teaching effect is established by using the multidimensional spatial hierarchical depth information mining method. Combined with spatial resolution parameter analysis, the image data feature detection method and the pixel division method are adopted to analyze the object model of medical image multimedia courseware teaching effect [15]. Then, we establish the spatial detail level parameter analysis model of medical image multimedia courseware-assisted teaching effect, build the database platform of medical image multimedia courseware-assisted teaching effect evaluation system through the parameter analysis of the spatial statistics model, and realize the bus transmission control of medical image multimedia courseware-assisted teaching effect evaluation system by using uniform resource locator SIP. Based on ORACLE, MYSQL, and other professional database processing tools, the information visualization reconstruction of the medical image multimedia courseware-assisted teaching effect evaluation system is realized, and we get the multilayer interactive functional component realization process of the system as shown in Figure 4.

According to the component design of Figure 4, the development platform of the medical image multimedia courseware-assisted teaching effect evaluation system is established in an embedded ARM environment [16], and the bottom control module of the medical image multimedia courseware-assisted teaching effect evaluation system adopts the integrated information interactive control method to construct the big data statistical data set of medical image multimedia courseware-assisted teaching effect evaluation, as shown in Table 1.

## 4. Evaluation and Optimization of Multimedia Courseware-Assisted Teaching Effect of Medical Images

### 4.1. Analysis of Constraint Characteristics of Medical Imaging Multimedia Courseware-Assisted Teaching Effect Evaluation

Based on the prediction of spatial attribute parameters, the classification big data mining model of medical image multimedia courseware-assisted teaching is constructed by using the deep learning algorithm with constraint index parameters such as courseware design appreciation, multimedia courseware theory, diversity of teaching methods, and discipline construction requirements, and the association rules and frequent item sets that can dynamically reflect the quality of medical image multimedia courseware-assisted teaching are mined [17, 18]. According to the spatial characteristics and attribute characteristics of medical image multimedia courseware-assisted teaching distribution, the statistical data analysis model of medical image multimedia courseware-assisted teaching effect is established, and the utilization rate of medical image multimedia courseware-assisted teaching effect is obtained based on spatial statistical analysis. The statistical dataset of medical image multimedia courseware-assisted teaching effect can be represented as

(1) $$\begin{array}{c} \Omega =\left\{\begin{array}{cc} \overset{⟶}{x}\in s|g_{j}\left(\overset{⟶}{x}\right)\leq 0, & j=1,\ldots ,l;\\ h_{j}\left(\left(\overset{⟶}{x}\right)\right.=0, & j=l+1,\ldots ,p \end{array}\right\}. \end{array}$$

In formula (1), $\overset{⟶}{x}$ represents the feature distribution set traversed by the global image, and *s* represents the comprehensive semivariance distribution neighborhood. $g_{j}\left(\overset{⟶}{x}\right)$ represents the statistical sample information of the *j* quantitative evaluation point, *l* represents the characteristic value of the attribute space control variable, $h_{j}\left(\overset{⟶}{x}\right)$ represents the best attribute parameter jump value, and *p* is the local variance of the multimedia image. Based on the constraint index parameters such as courseware design appreciation, multimedia courseware theory, diversity of teaching methods, and discipline construction requirements, a threshold analysis model of medical image multimedia courseware-assisted teaching is established by using image regional feature analysis [19, 20]. The difference factor under the constraint of the optimal utilization ratio of multimedia courseware for medical images is obtained. Through nonspatial data fusion cluster analysis and comprehensive semivariance feature estimation, the analytical model of optimal spatial attribute parameters is established, which improves the reliability of the evaluation of multimedia courseware for medical images [21, 22]. A feature matching model of medical image multimedia courseware-assisted teaching resource management is established, and the statistical feature quantity of medical image multimedia courseware-assisted teaching effect evaluation is obtained as follows:

(2) $$\begin{array}{c} Q=\frac{C_{1}\sum_{i=1}^{k}\exp\left[-S_{2}{\left(V_{i}-\mu \right)}^{2}\right]}{1+\text{exp}\left[-S_{1}\sum_{i=1}^{k}w_{i}\left(T_{i}-V_{i}\right)\right]}+\frac{y_{j}^{T}S_{b}y_{j}}{\lambda_{j}}. \end{array}$$

In formula (2), *C*_1_ and *S*_1_ are all multimedia feature classification sets of medical image multimedia courseware-assisted teaching resources management. Through subspace clustering, medical image multimedia courseware-assisted teaching resources are fused. The parameter constraint model is [0, 0.43, 0.15, 0.64, and 1], which indicates the recommendation degree of medical image multimedia courseware-assisted teaching information resources, and the semantic similarity is obtained as follows:

(3) $$\begin{array}{c} \;Z_{2}=\sum_{w\in W}{\hat{q}}^{w}\left(p_{I}-\gamma \hat{\theta }-Kr\right). \end{array}$$

In formula (3), $\hat{\theta }$ indicates the global equilibrium degree of medical image multimedia courseware-assisted teaching effect evaluation; *α* is a constant, and $\hat{\theta }$ indicates the fuzziness of medical image multimedia courseware-assisted teaching resources. Based on the prediction of spatial attribute parameters, the classification big data mining model of medical image multimedia courseware-assisted teaching is constructed by using a deep learning algorithm, and the association rules and frequent item sets that can dynamically reflect the quality of medical image multimedia courseware-assisted teaching are mined so as to realize the quality detection of medical image multimedia courseware-assisted teaching [23].

### 4.2. Quantitative Evaluation of Medical Multimedia Courseware-Assisted Teaching Effect

Based on the method of spatial and attribute parameter prediction, a dynamic constraint parameter model of medical image multimedia courseware-assisted teaching effect evaluation is established. Combined with subspace fusion cluster analysis, the maximum tree bifurcation method is adopted to conduct data-driven and segmentation scale adaptive estimation in the process of medical image multimedia courseware-assisted teaching effect evaluation. According to the spatial characteristics and attribute characteristics, the estimated construction effect of medical image multimedia courseware-assisted teaching is obtained, *A* = {*a*_1_, *a*_2_,…, *a*_*n*_} and *b* = {*b*_1_, *b*_2_,…, *b*_*m*_}. According to the above, the standard function of the teaching constraint index parameter is obtained as follows:

(4) $$\begin{array}{c} \left\{\begin{array}{c} \dot{x}=-\sigma x+\sigma y,\\ \dot{y}=-xz+rx-y,\\ \dot{z}=xy-bz. \end{array}\right. \end{array}$$

In formula (4), *x* represents the lateral component of the constraint index parameters of medical image multimedia courseware, *Y* represents the central component of the constraint index parameters of medical image multimedia courseware, *Z* represents the three-dimensional characteristic quantity of the constraint index parameters of medical image multimedia courseware, and *σ* represents the fuzzy membership parameter. Based on the machine learning algorithm, data from multiple data sources are merged together to obtain the grouping detection model as follows:

(5) $$\begin{array}{c} d_{i}=\sqrt{x_{i}^{2}+y_{i}^{2}+z_{i}^{2}}. \end{array}$$

In formula (5), *x*_*i*_ is the integration parameter of the *i*-th medical image multimedia courseware-assisted teaching distribution block, *y*_*i*_ is the auto-correlation characteristic matching coefficient of medical image multimedia courseware-assisted teaching, and *z*_*i*_^2^ is the fuzzy dynamic detection parameter. The entropy evaluation model of medical image multimedia courseware-assisted teaching effect evaluation is established, and the maximum information entropy distribution is as follows:

(6) $$\begin{array}{c} E_{\text{Snake}}=\sum_{0}^{N-1}\left[E_{\mathrm{int}}\left(vi\right)+E_{ext}\left(vi\right)\right]. \end{array}$$

In formula (6), *E*_int_(vi) represents the self-adaptive estimation parameter value of multimedia courseware-assisted teaching effect construction of medical images, *E*_ext_(vi) represents the local equation of multimedia courseware-assisted teaching images of medical images, and *N* represents the sample number of segmented patches. By using the method of fuzzy information fusion, the fuzzy clustering function of multimedia courseware-assisted teaching effect evaluation of medical images is expressed as follows:

(7) $$\begin{array}{c} \min\overset{⟶}{y}=\overset{⟶}{f}\left(\left(\overset{⟶}{x}\right)=\left(f_{1}\left(\overset{⟶}{x}\right),f_{2}\left(\overset{⟶}{x}\right),\ldots ,f_{m}\left(\overset{⟶}{x}\right)\right.\right). \end{array}$$

In formula (7), $\overset{⟶}{x}=\left(x_{1},x_{2},\ldots ,x_{n}\right)\in X\subset {ℜ}^{n}$ represents the abnormal error of elevation; *X* represents the level residual error of the utilization efficiency of multimedia courseware for medical images; $\;\overset{⟶}{y}\in Y\subset {ℜ}^{m}$ is the characteristic component representing the abnormal difference of medical image; *Y* represents the frequency quantization characteristic parameter value. Then, we calculate the variation function value of the medical image multimedia courseware-assisted teaching subblock, extract the statistical feature quantity of the medical image multimedia courseware-assisted teaching effect constraint index dataset by inverse feature analysis, and get the clustering model of medical image multimedia courseware-assisted teaching effect evaluation by fuzzy clustering maximum tree algorithm analysis. Under the optimized control rules, we establish the sparse scattered point parameter fusion model of medical image multimedia courseware-assisted teaching constraint index parameters, combining the analysis of generalized association rules and periodic association rules to realize the item set analysis of medical image multimedia courseware, and the statistical characteristic quantity of dynamic evaluation effectiveness is as follows:

(8) $$\begin{array}{c} E\left[N_{kl}^{*}N_{nm}\right]=\sigma^{2}\delta_{\text{km}}\delta_{\text{ln}}. \end{array}$$

In formula (8), *σ* is the root mean square error of minimum support, *δ*_km_is the regression steady-state parameter of medical image multimedia courseware aided teaching evaluation, and it is the joint detection probability density. The transaction database is transformed into a transaction matrix, and the fuzzy retrieval and information clustering analysis of constraint index parameters of medical image multimedia courseware are carried out through the feature extraction results [24, 25]. To sum up, the adaptive improved machine learning model is adopted to realize the classified guidance and teaching evaluation of medical imaging multimedia courseware [26, 27]. The implementation process is shown in Figure 5.

According to Figure 5, after inputting the dataset of medical image multimedia courseware auxiliary teaching effect evaluation, the medical image multimedia courseware auxiliary teaching effect is finally obtained through convergence judgment, and the final evaluation result is output to complete the research of medical image multimedia courseware auxiliary teaching effect evaluation based on the deep learning algorithm.

## 5. Simulation Test

In order to verify the classification guidance and teaching evaluation of medical image multimedia courseware, this paper analyzes and tests the parameters of medical image multimedia courseware with SPSS 22.0 Chinese version statistical analysis software and MATLAB simulation tools. First, the minimum confidence of medical image multimedia courseware classification is set at 43%, and the sample sequence size is 2400, and the rationality of course content design, classroom atmosphere, diversity of teaching methods, penetration of subject theory, and feedback benefit of classroom teaching are taken as explanatory variables.  Table 2 shows the distribution of descriptive statistical analysis results of explanatory variables.

The low point of constraint dynamic frequency of medical multimedia courseware is 54 Hz, the sampling rate of association rules is 26 kHz, and the length of classification data of medical multimedia courseware is 12,000 cm. Thus, the distribution of big data statistical characteristics of medical multimedia courseware is shown in Figure 6.

Taking the data of Figure 7 as the research object, the multimedia courseware of medical images is used to assist in teaching and data clustering, and the output is shown in Figure 7.

According to the analysis of Figure 7, this method can effectively realize the dynamic evaluation of multimedia courseware for medical images, improve the clustering performance of constraint index parameters of multimedia courseware for medical images, and test the storage cost after the evaluation of talent cultivation quality, as shown in Figure 8.

According to the analysis of Figure 8, the method in this paper compares the reliability of medical image multimedia courseware-assisted teaching evaluation, and the reliability results are all above 90%, with good performance.

## 6. Conclusions

This paper presents a method of evaluating the effect of medical image multimedia courseware based on the deep learning algorithm to realize the quantitative evaluation of the teaching effect of medical image multimedia courseware and to improve the teaching quality of medical image courses. The simulation test shows the superior performance of this method in improving the evaluation ability of medical image multimedia courseware-assisted teaching, which is shown in the following aspects:

1. This method has important significance in improving the quality of medical image multimedia courseware-assisted teaching
2. The effect evaluation of medical image multimedia courseware based on the deep learning algorithm can achieve effective clustering output
3. In this paper, the reliability of medical image multimedia courseware-assisted teaching evaluation was compared, and the results were above 90%

## Figures and Tables

**Figure 1:** Deep learning model with multiple hidden layers.

**Figure 2:** Overall system architecture.

**Figure 3:** Network design of the system.

**Figure 4:** Implementation process of functional components of multilayer interaction.

**Figure 5:** Implementation process of the improved algorithm.

**Figure 6:** Time-domain distribution of constraint index parameters of medical image multimedia courseware-assisted teaching effect evaluation. (a) Test sample. (b) Training sample. (c) Statistical sequence sample of medical image multimedia courseware effect evaluation.

**Figure 7:** Cluster output of multimedia courseware of medical images for assisting teaching evaluation.

**Figure 8:** Comparative test of evaluation reliability.

**Table 1:** Big data statistical data set of medical imaging multimedia courseware-assisted teaching effect evaluation.

Sample group of medical multimedia courseware resources	Test sample sequence	Model parameter	Constraint factor
Test set 1	8560	5.409	0.922
Test set 2	5985	6.293	0.869
Test set 3	7999	2.964	0.629
Test set 4	3497	2.192	0.757
Test set 5	6983	1.455	0.697
Test set 6	4110	5.438	0.352
Test set 7	5484	8.611	0.015
Test set 8	5560	7.216	0.328
Test set 9	8902	1.212	0.260
Test set 10	3795	1.744	0.836
Test set 11	5374	6.497	0.737
Test set 12	9051	6.460	0.948
Test set 13	2425	4.410	0.718
Test set 14	6376	9.822	0.714

**Table 2:** Descriptive statistical analysis results of explanatory variables.

Explanatory variable	Equivocation	Value factor	Correlation	Statistical characteristic quantity
Rationality of course content design	0.039	0.159	0.336	0.8404
Classroom atmosphere	0.383	0.149	0.579	0.9557
Diversity of teaching methods	0.424	0.452	0.916	0.6674
Subject theoretical permeability	0.201	0.890	0.528	0.1089
Efficiency of classroom teaching feedback	0.438	0.651	0.655	0.2740

## Data Availability

The raw data supporting the conclusions of this article will be made available by the authors, without undue reservation.
